The article "Low expression of protocadherin7 (PCDH7) is a potential prognostic biomarker for primary non-muscle invasive bladder cancer" was published in 2016. Journal: Oncotarget.

# Low expression of protocadherin7 (PCDH7) is a potential prognostic biomarker for primary non-muscle invasive bladder cancer

**DOI:** 10.18632/oncotarget.8635

**Published:** 2016-04-07

**Authors:** Ying-Li Lin, Yan-Ling Wang, Xing-Li Fu, Wen-Ping Li, Yu-Hao Wang, Jian-Guo Ma

**Affiliations:** ^1^ Department of Urology, Xuzhou Cancer Hospital, Affiliated Xuzhou Hospital of Jiangsu University, Xuzhou, 221000, Jiangsu, China; ^2^ Department of Anesthesiology, Third Affiliated Hospital of Sun Yat-sen University, Guangzhou, 510630, Guangdong, China; ^3^ Health Science Center, Jiangsu University, Zhenjiang, 212000, Jiangsu, China; ^4^ Department of Urology, Third Hospital of Hebei Medical University, Shijiazhuang, 050051, Hebei, China; ^5^ Department of Clinical Medicine, Nanjing Medical University, Nanjing, 210000, Jiangsu, China

**Keywords:** bladder cancer, biomarker, protocadherin7, PCDH7, prognosis

## Abstract

Bladder cancer is a heterogeneous disease with outcome difficult to predict, and novel predictive biomarkers are needed. PCDH7, a member of protocadherins family, functions as tumor suppressor in several human cancers. The human PCDH7 gene is localized in chromosome 4p15, which is often inactivated in human cancers, including bladder cancer. The aim of this study was to investigate the clinical significance of PCDH7 expression in non-muscle invasive bladder cancer (NMIBC). PCDH7 expression was examined using immunohistochemical staining in 199 primary NMIBC tissues and 25 normal bladder epithelial tissues. Then the relationship between PCDH7 expression and clinicopathologic features was evaluated. Kaplan-Meier survival analysis and Cox analysis was used to evaluate the correlation between PCDH7 expression and prognosis. PCDH7 expression in NMIBC tissues was significantly lower than that in normal bladder epithelial tissues (*P* < 0.001). Low PCDH7 expression correlated with advanced grade (*P* = 0.021) and larger tumor size (*P* = 0.044). Moreover, patients with low PCDH7 expression have shorter recurrence-free survival (*P* < 0.001), progression-free survival (*P* = 0.007) and overall survival (*P* = 0.011) than patients with high PCDH7 expression. Low PCDH7 expression is an independent predictor of recurrence-free survival (multivariate Cox analysis: *P* = 0.007), progression-free survival (multivariate Cox analysis: *P* = 0.014) and overall survival (multivariate Cox analysis: *P* = 0.004). The findings indicate that low PCDH7 expression is a potential prognostic biomarker for primary NMIBC.

## INTRODUCTION

Bladder cancer is a common disease worldwide [1, 2]. Moreover, it's a heterogeneous disease with outcome difficult to predict [3, 4]. Bladder cancer can be divided into two groups: non-muscle invasive bladder cancer (NMIBC) and muscle invasive bladder cancer (MIBC), based on histopathology and clinical behaviors [5]. NMIBC represents over 70% of all newly diagnosed bladder cancer cases, and approximately 90% are transitional cell carcinoma in histology. Currently, transurethral resection of bladder tumor (TURBT) is the main treatment for NMIBC. Unfortunately, approximately 70% of NMIBC will relapse and 15% will progress to MIBC after TURBT [6, 7]. Current risk scores based on traditional clinical and pathological parameters can provide important but limited prognostic information, and novel reliable biomarkers are needed to predict patients’ outcome [8–10].

PCDH7 is a member of protocadherins (PCDHs) family, belonging to cadherin superfamily. The human PCDH7 gene is localized in chromosome 4p15, which encodes the membrane protein that is believed to function in cell-cell recognition, adhesion and signal transduction [11]. The protocadherin family can be classified into two groups: clustered PCDHs (PCDH α, β and γ family) and non-clustered PCDHs (PCDH1, 7, 8, 9, 10, 11, 12, 15, 16, 17, 18, 19, 20, 21 and MUCDHL), based on their genomic structure [11]. Recent researches suggest that non-clustered PCDHs can increase cell-cell adherin and other molecules’ function. Moreover, some non-clustered PCDHs have been suggested as candidate tumor suppressor genes in human tumors, including PCDH7, 8, 9 and 21 etc [11–13]. PCDHs are often silenced by DNA methylation in human cancers [11]. Recent studies indicated that PCDH7 is frequently inactivated by DNA methylation in bladder cancer and functions as a tumor suppressor [14]. However, its prognostic value in bladder cancer needs to be further elucidated.

To our knowledge, no study has evaluated the prognostic role of PCDH7 expression in bladder cancer. The aim of this study was to evaluate the impact of PCDH7 expression on clinicopathological parameters and prognosis in NMIBC patients.

## RESULTS

### PCDH7 expression in NMIBC tissues and normal bladder epithelial tissues

The expression of PCDH7 was examined in 199 NMIBC tissues and 25 normal bladder epithelial tissues using immunohistochemical staining (Table 1). High PCDH7 expression was detected in all of the normal bladder epithelial tissues (100%). While high PCDH7 expression was only detected in 84 (42.2%) patients with primary NMIBC (Figure 1). PCDH7 expression was lower in NMIBC tissues than that in the controls and the difference was statistically significant (*P* < 0.001).

**Table 1:** The clinical and pathological features of NMIBC patients (n = 199)

Features	Variables	No. (%)
Age (years)	≤ 65	74 (37.2)
	> 65	125 (62.8)
Sex	Male	138 (69.3)
	Female	61 (30.7)
Tumor size (cm)	≤ 3	109 (54.8)
	> 3	90 (45.2)
Tumor number	Single	114 (57.3)
	Multiple	85 (42.7)
Grade	G1	70 (35.2)
	G2	65 (32.7)
	G3	64 (32.1)
Stage	Ta	72 (36.2)
	T1	127 (63.8)
Recurrence	Yes	71 (35.7)
	No	128 (64.3)
Progression	Yes	21 (10.6)
	No	178 (89.4)
Death	Yes	23 (11.6)
	No	176 (88.4)

**Figure 1:** Representative PCDH7 expression in normal bladder epithelial tissues and NMIBC tissues (× 400) High expression: (**A**) (normal bladder epithelial tissue) and (**B**) (NMIBC); Low expression: (**C**) (NMIBC) and (**D**) (NMIBC).

### Association between PCDH7 expression and clinicopathologic parameters in NMIBC patients

The association between PCDH7 expression and clinicopathologic parameters was assessed, as shown in Table 2. The results indicated that low PCDH7 expression correlated with advanced grade (*P* = 0.021) and larger tumor size (*P* = 0.044). However, no significant association was observed between PCDH7 expression and age (*P* = 0.157), sex (*P* = 0.243), pathologic stage (*P* = 0.631) or tumor number (*P* = 0.799).

**Table 2:** Association between PCDH7 expression and clinicopathologic features in NMIBC patients (n = 199)

Features	Variables	No. (%)	PCDH7 Expression		*P*
			High	Low	
Age (years)	≤ 65	74 (37.2)	36 (48.6)	38 (51.4)	0.157
Sex	> 65	125 (62.8)	48 (42.2)	77 (57.8)	
Tumor size (cm)	Male	138 (69.3)	62 (44.9)	76 (55.1)	0.243
Tumor number	Female	61 (30.7)	22 (36.1)	39 (63.9)	
Grade	≤ 3	109 (54.8)	53 (48.6)	56 (51.4)	0.044
Stage	> 3	90 (45.2)	31 (34.4)	59 (65.6)	
	Single	114 (57.3)	49 (43.0)	65 (57.0)	0.799
	Multiple	85 (42.7)	35 (41.2)	50 (58.8)	
	G1	70 (35.2)	35 (50.0)	35 (50.0)	0.021
	G2	65 (32.7)	31 (47.7)	34 (52.3)	
	G3	64 (32.1)	18 (28.1)	46 (71.9)	
	Ta	72 (36.2)	32 (44.4)	40 (55.6)	0.631
	T1	127 (63.8)	52 (40.9)	75 (59.1)	

### Association between PCDH7 expression and recurrence-free survival in patients with NMIBC

Kaplan-Meier analysis and log-rank test indicated that patients with low PCDH7 expression had worse outcome than patients with high PCDH7 expression (*P* < 0.001; Figure 2). To identify the prognostic value of PCDH7 expression for recurrence-free survival, univariate and multivariate Cox analysis was conducted. The results confirmed that low PCDH7 expression of is an independent prognostic factor for recurrence-free survival of patients with NMIBC (univariate Cox analysis, Exp (B): 3.977; 95% CI: 1.603–7.173; *P* = 0.000. multivariate Cox analysis, Exp (B): 3.251; 95% CI: 1.364–6.172; *P* = 0.007. Table 3).

**Figure 2:** Associations between PCDH7 expression and recurrence-free survival of NMIBC patients Patients with low expression of PCDH17 showed significantly shorter recurrence-free survival than those with high expression of PCDH17. (log-rank test, *P* < 0.001).

**Table 3:** The prognostic value of low expression of PCDH7 for the recurrence-free survival in univariate and multivariate Cox regression analysis

Varivale	Univariate analysis			Multivariate analysis		
	Exp (B)	95% CI	*P*	Exp (B)	95% CI	*P*
Age	0.965	0.962–2.547	0.642			
Sex	1.055	0.743–3.421	0.254			
Tumor size	2.137	0.936–3.459	0.043	1.254	0.768–3.251	0.137
Tumor number	1.784	0.895–4.214	0.086			
Grade	3.173	1.238–5.8974	0.009	2.147	1.139–5.026	0.017
Stage	2.581	1.066–4.763	0.035	1.468	0.932–4.297	0.079
PCDH7 expression	3.977	1.603–7.173	0.000	3.251	1.364–6.172	0.007

### Association between PCDH7 expression and progression-free survival in patients with NMIBC

To further investigate the association between PCDH7 expression and progression-free survival, Kaplan-Meier analysis and log-rank test was performed according PCDH7 expression. The result indicated that low PCDH7 expression was significant associate with worse progression-free survival of the patients (*P* = 0.007; Figure 3). Moreover, univariate and multivariate Cox analysis suggested that low expression of PCDH7 is an independent predictor for the progression-free survival of NMIBC patients (univariate Cox analysis, Exp (B): 4.381; 95% CI: 1.731–8.542; *P* = 0.006. multivariate Cox analysis Exp (B): 3.428; 95% CI: 1.547–6.781; *P* = 0.014. Table 4).

**Figure 3:** Associations between PCDH7 expression and progression-free survival of NMIBC patients Patients with low expression of PCDH17 showed significantly shorter progression-free survival than those with high expression of PCDH17. (log-rank test, *P* = 0.007).

**Table 4:** The prognostic value of low expression of PCDH7 for the progression-free survival in univariate and multivariate Cox regression analysis

Varivale	Univariate analysis			Multivariate analysis		
	Exp (B)	95% CI	*P*	Exp (B)	95% CI	*P*
Age	1.047	0.796–5.384	0.469			
Sex	0.985	0.864–3.142	0.576			
Tumor size	1.264	0.836–2.397	0.135			
Tumor number	1.724	0.695–6.453	0.054			
Grade	2.522	1.034–4.643	0.027	1.453	1.326–3.542	0.044
Stage	3.051	1.136–5.643	0.013	2.253	1.53–4.937	0.032
PCDH7 expression	4.381	1.731–8.542	0.006	3.428	1.547–6.781	0.014

### Association between PCDH7 expression and overall survival in patients with NMIBC

The five-year overall survival data were available form all the NMIBC patients. For patients with low PCDH7 expression had worse outcome than patients with high PCDH7 expression (*P* = 0.011; Figure 4). In addition, Cox analysis indicated that low expression of PCDH7 is independently associated with poor overall survival. The result of univariate (Exp (B): 3.466; 95% CI: 1.382–9.431; *P* = 0.013) and multivariate (Exp (B): 3.215; 95% CI: 1.463–10.776; *P* = 0.004) Cox analysis was shown in Table 5.

**Figure 4:** Associations between PCDH7 expression and five-year overall survival of NMIBC patients Patients with low expression of PCDH17 showed significantly shorter overall survival than those with high expression of PCDH17. (log-rank test, *P* = 0.011).

**Table 5:** The prognostic value of low expression of PCDH7 for the five-year overall survival in univariate and multivariate Cox regression analysis

Varivale	Univariate analysis			Multivariate analysis		
	Exp (B)	95% CI	*P*	Exp (B)	95% CI	*P*
Age	0.891	0.674–6.346	0.785			
Sex	1.033	0.855–5.253	0.462			
Tumor size	1.943	0.766–8.467	0.116			
Tumor number	1.783	0.705–14.306	0.147			
Grade	2.274	1.241–7.842	0.037	2.042	0.785–13.692	0.127
Stage	3.783	1.523–8.437	0.008	2.447	1.311–6.016	0.017
PCDH7 expression	3.466	1.382–9.431	0.013	3.215	1.463–10.776	0.004

## DISCUSSION

Bladder cancer is a common disease worldwide, and the morbidity is increased progressively [15, 16]. Simultaneously, it's a complex and heterogeneous disease, leading to extremely different clinical behaviors and outcomes [17]. Recurrence and progression is the main character of NMIBC. The main challenge in clinical practice is to distinguish aggressive tumors from indolent ones [8, 18–20]. Currently, clinical and pathological factors are used as predictors, but they fail to assess patients’ outcome accurately. Thus, more work is required to identify reliable, convenient and cost-effective predictors [8, 17]. Immunohistochemical staining is a widely used technique. In this study we used this method to assess the expression of PCDH7 in NMIBC and then evaluated its clinical significance. We are hoping to establish an accurate predictor which can be used in clinical routinely.

Recent studies suggested that PCDH7 functions as a tumor suppressor in human cancers. Bujko et al. identified that PCDH7 expression was decreased in colorectal cancer, and the same finding was also occurred in lung cancer [21, 22]. DNA methylation is one of the most common epigenetic changes, inducing the inactivation of gene expression [23]. Beukers et al. indicated that PCDH7 was hypermethylated frequently in bladder cancer [24]. These findings promote us to investigate the clinical significance of PCDH7 expression in bladder cancer.

The main findings of the present study are as following three points. First, PCDH7 expression was decreased in NMIBC tissues. Second, low PCDH7 expression was significantly associated with high grade, tumor recurrence and progression after curative surgery. Third, low PCDH7 expression was significantly associated with the poor outcome of the patients. In support of this, recurrence-free survival, progression-free survival and overall-survival was evaluated separately. Kaplan-Meier analysis and log-rank test indicated that patients with low PCDH7 expression had worse recurrence-free survival, progression-free survival and overall-survival than patients with high PCDH7 expression. The result suggested that low PCDH7 expression is a predictor for the poor prognosis. To further evaluate its predictive value, Cox proportional hazard model was performed. Interestingly, univariate and multivariate analysis demonstrated that low PCDH7 expression is an independent predictor for the poor outcome. Our findings suggested low PCDH7 expression is a potential prognostic biomarker for NMIBC patients.

A key strength of this study was that only primary NMIBC patients were included. As bladder cancer is a heterogeneous disease, evaluating the effectiveness of a gene expression as predictor within the homogeneous group is very important. For bladder cancer patients, the expression of PCDH7 in tumor tissues should be detected after surgery. For patients with low PCDH7 expression, the surveillance strategy should be strengthen and more aggressive adjuvant therapy should be performed after initial curative surgery, so as to achieve better prognosis. Our finding may help in establishing individualized therapy strategy. Our study also has some limitations. The sample size is not larger enough, and this study was performed in one center. Future multi-center studies with larger sample size are needed to confirm our findings, before it is used routinely in clinical practice.

In conclusion, we reported for the first time that PCDH7 expression was decreased in NMIBC tissues and low PCDH7 expression was associated high pathologic grade, tumor recurrence and progression. Moreover, low PCDH7 expression is an independent prognostic factor for the outcome of NMIBC patients.

## MATERIALS AND METHODS

### Patients and tissue samples

This study was performed according to the Declaration of Helsinki and was approved by the ethics committee of Third Hospital of Hebei Medical University (HMU20020707X). Informed written consent was obtained from all the participants. A total of 224 tissues were collected in this study, including 199 primary NMIBC tissues obtained from patients who underwent TURBT and 25 normal bladder epithelial tissues obtained from benign prostatic hyperplasia patients (median age 65, range 52–78) who underwent transurethral resection of prostate at Third Hospital of Hebei Medical University, between 2003 and 2009. None of the NMIBC patients had received chemotherapy or radiation therapy before the surgery. All specimens were fixed in 10% formalin and embedded in paraffin. Hematoxylin and eosin stained slides were evaluated by two senior pathologists who blinded to the patients’ clinical information.

The tumor grade and stage were defined according to the criteria of the WHO (1973) and the TNM classification of the International Union Against Cancer (UICC, 2002) [25, 26]. A second TUR was performed 2–4 weeks after initial surgery if a high-grade tumor was detected. Patients with intermediate or high risk NMIBC were given one cycle of intravesical instillation therapy, and all the patients were followed up and managed according to standard guidelines [27, 28]. Recurrence was defined as the return of NMIBC at a lower or equivalent pathologic stage, and progression was defined as muscle invasion or lymph node/distant metastatic disease [29].

### Immunohistochemistry

Immunohistochemical staining was performed as reported previously [30]. Briefly, formalin fixed and paraffin embedded specimens in 4-um thick sections were deparaffinized in xylene, and xylene was removed through a serious of alcohols. Endogenous peroxidase activity was blocked with 3% H_2_O_2_ for 10 min. Antigen retrieval was performed in boiling citrate buffer for 15 min. After that the sections were incubated with mouse antihuman PCDH7 antibody (SC-517042; Santa Cruz Biotechnology Inc., Santa Cruz, Calif., USA) at a 1:100 dilution at 4°C overnight. After washing with PBS, sections were incubated with second antibody (PV-9001; Beijing ZhongShan, China) at 37°C for 20 min and washed 3 times with PBS. Finally, the reactions were developed with 3, 3′-diaminobenzidine (ZLI-9017; Beijing ZhongShan, China), and all sections were counterstained with hematoxylin. PCDH7 expression of positive cells was defined as PCDH7 staining observed around the cell membranes. The percentage of positive cells was calculated by dividing the total number of bladder epithelial cells in at least ten randomly chosen non-overlapping high-power fields for each case. The PCDH7 expression result was evaluated by two senior pathologists in our center who blinded to the survival data. PCDH7 expression levels were classified semi-quantitatively combining the proportion and intensity of positively stained immunoreactive cells. The percentage of positive-staining tumor cells was scored as follows: 0 (< 5% positive tumor cells); 1 (5%–50% positive tumor cells); and 2 (> 50% positive tumor cells). Staining intensity was scored as follows: 0 (no staining or only weak staining); 1 (moderate staining); and 2 (strong staining). The sum of the staining intensity score and the percentage score was used to define the PTK7 protein expression levels: 0–2, low expression and 3–4, high expression [31].

### Statistical analysis

The difference of PCDH7 expression between NMIBC patients and controls were evaluated using Fisher's exact test. The correlation between PCDH7 expression and clinicopathologic features was evaluated by chi-square test. Survival curves were plotted using the Kaplan-Meier method and log-rank test. The Cox proportional hazard model was used for the univariate and multivariate analysis of the prognostic factors for recurrence-free survival, progression-free survival and overall survival. The statistical analyses were performed using the SPSS 16.0 software (SPSS, Chicago, IL, USA). *P* < 0.05 was considered to be statistically significant.
